# Effects of Combining Cognitive Behavioral Therapy with Bilateral Upper Limb Training in Stroke Patients: A Randomized Controlled Trial

**DOI:** 10.1155/2022/4688113

**Published:** 2022-07-07

**Authors:** SoEun Choi, DeokJu Kim

**Affiliations:** ^1^Department of Occupational Therapy, Cheongju St. Mary's Hospital, Cheongju, Republic of Korea; ^2^Department of Occupational Therapy, College of Health & Medical Sciences, Cheongju University, Cheongju, Republic of Korea

## Abstract

CBT has a beneficial effect on depression and anxiety; however, the number of cases where therapy was used in patients with stroke was rare. In addition, there is still a lack of research on the effects of occupation-based training and the effects of bilateral upper limb training that provides an intervention based on patients' state of hemiplegic upper limb function. This study investigated the effects of combining CBT and occupation-based bilateral upper limb training on the depression, anxiety, upper limb function, and occupational performance. The experimental group was given 30-min cognitive behavioral therapy and occupation-based bilateral upper limb training, while the control group was given 30-min conventional occupational therapy and occupation-based bilateral upper limb training. For both groups, the intervention was given as a 30-min session once a day and five times a week for 4 weeks. Following intervention, the experimental group showed significant within-group variance for automatic thoughts, depression, anxiety, upper limb function, and occupational performance only (*p* < 0.01). For between-group variance, a significant difference was found for automatic thoughts, depression, anxiety, and occupational performance (*p* < 0.01), however, not for upper limb function (*p* > 0.05). In this study, it is meaningful that this author provided good guidelines for therapists and caregivers by organizing and providing actual programs in a very rare situation where cognitive behavioral therapy was applied to stroke patients.

## 1. Introduction

Stroke reduces brain function and causes severe conditions such as linguistic, cognitive, or emotional impairment [1]. In a study, it was found that stroke hospitalized patients were highly dependent on activity of daily living (ADL) and experienced high fatigue on instrumental activity of daily living (IADL) [2]. Of note is the limiting impact on the performance of ADL requiring functional manipulation of the upper limbs such as eating, getting dressed, personal hygiene, grooming, bathing, toilet sanitation, managing personal articles, social activities, transport between communities, and managing personal affairs [3, 4]. In another study, upper limb dysfunction caused by hemiplegia has a very negative effect on ADL, so it is reported that rehabilitation treatment that promotes an independent life after stroke is important [5].

Occupation-based bilateral upper limb training provides the patients tasks resembling ADL where bilateral upper limb function is required, to induce active participation and motivation and to improve the occupational performance, leading to functional recovery and independence [6]. Over 80% of occupational therapy is conducted in a hospital setting in South Korea and focused mostly on functional recovery due to time or environmental limitation [7]. The effects of occupation-based bilateral upper limb training reflecting the state of hemiplegic upper limbs must be investigated.

Patients with stroke experience not only physical dysfunction but also reduced drive or vigor caused by mood disturbances such as stress from unnatural appearance, maladjustment to unfamiliar hospital environment, or anxiety about future return to society. Previous studies on the psychosocial state of patients with stroke reported anxiety and depression as the main psychological problems, while the conditions were experienced by 23% and 19%, respectively, of early stroke patients within 6 months of onset [8]. The main psychological problem experienced by patients with depression is anxiety, and the reported causes of psychological anxiety include poststroke physical dysfunction, personality change, and emotional trauma [9].

The best-known intervention for depression and anxiety is cognitive behavioral therapy (CBT). The emphasis in CBT is placed on cognitive restructuring that turns negative thoughts and beliefs of the stroke incidence into more positive ones, based on the view that the cognition and interpretation of the events that occur in a person's life affect the person's emotion and behavior [10–14]. The form of group counseling was reported to reduce depression in the elderly at a care facility [15], and the effect of reducing anxiety and negative thoughts was reported in undergraduate students with social anxiety, in whom dysfunctional beliefs were changed [16].

CBT has a beneficial effect on depression and anxiety; however, the number of cases where therapy was used in patients with stroke was rare. Some studies have investigated the effects of occupation-based training that leads patients to set a personal goal for a desired activity to increase rehabilitation motivation and presents tasks that resemble actual daily activities or the effects of bilateral upper limb training that provides an intervention based on patients' state of hemiplegic upper limb function.

This study investigated the effects of combining CBT and occupation-based bilateral upper limb training on the depression, anxiety, upper limb function, and occupational performance.

## 2. Methods

### 2.1. Participants

This study recruited 20 patients with stroke receiving inpatient treatment at C General Hospital and I Rehabilitation Clinic located in Cheongju-si, from June to September 2020. The inclusion criteria were patients diagnosed by a specialist after 3 months from the date of onset and with a Brunnstrom recovery stage (BRS) ≥3 for proximal and distal parts of the hemiplegic upper limb while being able to write without verbal communication. The exclusion criteria were patients with a history of stroke or a neurological or surgical disease, those with a recent experience of a clinical study on rehabilitation or drug administration, those with repeating seizures during the period of treatment or a severe damage to vision, and who were on drugs for improving rigidity.

### 2.2. Study Design

This study was conducted as a randomized controlled study using computerized randomization. It used a single-blind design to prevent participants from knowing the group they belonged to. Before the study, the approval of the Cheongju University Institutional Review Board (IRB No. 1041107-202006-HR-030-01) was obtained, and a written consent for participation was received from all participants given the explanation of the purpose and contents of the study. We used simple randomization to conduct a randomized controlled study. The participants were selected based on the results BRS, and the 20 participants who fulfilled the inclusion criteria were randomized between the experimental and control groups using a computer program. Before intervention, each participant selected a meaningful occupation involving a bilateral upper limb movement on their own via the Canadian Occupational Performance Measure (COPM). The experimental group received a 30-min session (10-min CBT and 20-min occupation-based bilateral upper limb training in the treatment room), five times a week for 4 weeks. The control group received a different 30-min session (10-min conventional occupational therapy of neurodevelopmental therapy, exercise therapy based on Bobath approach or proprioceptive neuromuscular facilitation, in-hand manipulation or dexterity training, followed by 20 min occupation-based bilateral upper limb training in the treatment room) five times a week for 4 weeks. All participants were unaware of which group they belonged to, and the study proceeded from pretest to intervention to posttest (Figure 1).

### 2.3. Cognitive Behavioral Therapy

The program used in this study for CBT comprised a course for cognitive restructuring where the participants searched for negative automatic thoughts and beliefs and turned them into positive ones on their own accord. The program contained self-reported worksheet activity, a behavioral training and the therapist's feedback, and verbal communication, based on the Learning Cognitive Behavior Therapy developed by Wright, Brown, Thase, and Basco and translated by Kim [17], the real-time CBT developed by McMullin and translated by Kim [14], and various previous studies regarding the effects of CBT [11, 13, 18–23]. The novel program was reviewed by two professors at the Department of Psychiatry who were occupational therapy specialists, then subsequently revised, and complemented before use. Stages 1–3 are the introductory phases where the participants are educated generally on stroke, CBT, and use of both hands in daily activities. Stages 4–17 are the development phases with the focus on step-by-step cognitive restructuring. The participants were guided to perform activities related to cognitive restructuring, while participating in the energization of behavior and relaxation training. Stages 18–20 are the wrap-up phases where the past sessions were reviewed, and the course was completed. The cognitive behavioral therapy was conducted only on the experimental group as a 10-min session with 20 sessions in total, five times a week for 4 weeks, preceding the bilateral upper limb training (Table 1).

### 2.4. Occupation-Based Bilateral Upper Limb Training

The occupation-based bilateral upper limb training used in this study comprised selected activities that can be performed in a hospital setting. The COMP was carried out to lead the participants to voluntarily select the occupation-based activities in an interview with a therapist where personal goals for the activities were set. The occupational therapy was conducted as a 1 : 1 session with a therapist with 3 or more years of experience, after selecting five most important occupations. Each selected activity was reviewed for suitability by the participant and the therapist together, and in the absence of problems, the therapy was continued. Throughout training, the therapist provided continuous feedbacks alongside instructions, while the participants performed the activities in accordance with the level of hemiplegia and based on the therapist's instructions for cases that could occur during the performance of the bilateral upper limb activity. Additionally, the materials or spatial arrangements necessary to perform the activities as they would be at home were prepared in advance through communication between the participant and the therapist. Participants were trained in both experimental and control groups as a 20-min session for 20 sessions, five times a week for 4 weeks.  Table 2 summarizes examples of intervention activities selected by the participants in the experimental group (Figure 2) (Table 2).

### 2.5. Measurements

#### 2.5.1. Negative Automatic Thoughts

To evaluate the negative automatic thoughts in stroke patients, the Automatic Thoughts Questionnaire-Negative (ATQ-N) was used. The tool comprised 30 questions on a five-point scale. The total score ranged between 30 and 150, and a higher score indicated a higher frequency of negative thoughts. The reliability of the tool was 0.94 [21].

#### 2.5.2. Depression

To evaluate changes in the depression level in stroke patients, the Korean Depression Scale (KDS) was used. The tool comprised 30 questions on a five-point scale with six subcategories: negative thoughts on the future, negative thoughts on the self, nervousness and restlessness, somatization symptoms, depressive feelings, and loss of drive. The total score ranged between 0 and 120, and a higher score indicated a higher level of depression. The reliability of the tool was 0.88 [24].

#### 2.5.3. Anxiety

To evaluate changes in the anxiety level, the State Trait Anxiety Inventory-Korean YZ (STAI-KYZ) was used. The tool tests state anxiety and trait anxiety, categorized for evaluation based on 20 questions on a four-point scale. The total score ranged between 20 and 80, and a higher score indicated a higher anxiety level. The reliability of the tool was 0.88 [25].

#### 2.5.4. Upper Limb Function

The changes in upper limb function were evaluated using two different tools. The first was Manual Function Test (MFT), comprising four items on upper limb movement, two items on grip strength, and two items on finger manipulation. A score of 1 was given to performance and 0 to nonperformance. The total score was the sum of the score of each item, with the maximum of 32 points, which was multiplied by 3.125 to be converted to 100 for recording. The reliability of the tool was 0.99 for the hemiplegic limb and 0.83 for the nonhemiplegic limb [26]. The second tool, Motor Activity Log (MAL), measured the use of the hemiplegic upper limb in daily activities. The tool comprised 30 items on various basic and instrumental daily activities that indicated the level of recovery of the hemiplegic upper limb. The intrarater reliability was 0.81–0.87, and the test-retest reliability was 0.91 [27].

#### 2.5.5. Occupational Performance

Changes in occupational performance were evaluated using the COPM. This semistructured tool allows the client to identify a problem in activity on their own. Each item on a 10-point scale indicates importance, and the intervention targets the top five occupations. Each target occupation is scored on a 10-point scale, to indicate the current performance and satisfaction. The test-retest reliability of the COPM is high, 0.65–0.80 for performance and 0.75–0.89 for satisfaction. In this study, the participants were led to set the goals by themselves, while the tool was used to compare the performance and satisfaction between pretest and posttest [28].

### 2.6. Data Analysis

The statistical analysis for all data in this study was performed using the SPSS version 24.0. The normality for the participants was tested using the Shapiro-Wilk test, and due to the absence of normality, the nonparametric statistics was used. The general characteristics of the participants were analyzed using the chi-squared test and the description statistics, and the functional homogeneity before the intervention was tested using the Mann–Whitney *U* test. The within-group and between-group differences between pretest and posttest were analyzed using the Wilcoxon signed rank test and the Mann–Whitney *U* test, respectively. The significance level was set to 0.05.

## 3. Results

### 3.1. Demographics and Baseline Characteristics

The experimental group consisted of seven male and three female patients, and the control group consisted of five male and five female patients. The average participant age was 61.40 (9.33) years in the experimental group and 66.60 (8.63) years in the control group. In both groups, the case type was infarction for six patients and hemorrhage for four patients, while the case period on average was 4.50 (1.17) months in the experimental group and 4.60 (1.17) months in the control group. The results showed no significant difference across all variables of general characteristics: age, sex, case type, hemiplegic side, case period, and BRS (*p* > 0.05) (Table 3).

### 3.2. Negative Automatic Thoughts, Depression, Anxiety, Upper Limb Function, and Occupational Performance

For ATQ-N, the experimental group showed a significant decrease (*p* < 0.01), while the control group showed no significant change (*p* > 0.05). For KDS, the experimental group showed a significant decrease (*p* < 0.01), while the control group showed no significant change (*p* > 0.05). For STAI-KYZ, the experimental group showed a fall in state and trait anxiety with significance (*p* < 0.01), while the control group showed no significant difference (*p* > 0.05). A significant difference was found for between-group variance regarding depression, anxiety, and in the negative automatic thoughts (*p* < 0.001). For MFT, both experimental and control groups showed a statistically significant improvement (*p* < 0.01), and for MAL, both the quantity and quality of motion showed a significant improvement in both experimental and control groups (*p* < 0.01). For COPM, a significant improvement was found for performance and satisfaction in both experimental and control groups (*p* < 0.01). No significant difference was found for between-group variance regarding upper limb function (*p* > 0.05), while the between-group variance regarding occupational performance showed a significant difference (*p* < 0.001) (Table 4).

## 4. Discussion

This study was conducted as a randomized controlled study to investigate the effects of combining CBT and occupation-based bilateral upper limb training in stroke patients regarding negative automatic thoughts, depression, anxiety, upper limb function, and occupational performance.

The CBT used in this study comprised a course towards cognitive restructuring where the participants searched for negative automatic thoughts and beliefs and turned them into positive ones on their own accord. Based on the literature introducing the CBT [14, 17] and various previous studies [11, 13, 18–22], the present study proceeded with a worksheet activity for cognitive restructuring, a behavioral training, and the therapist's feedbacks. The participants were requested to complete two worksheets for each session of the course: (i) a log to record the events of the day and the negative automatic thoughts and feelings upon a particular event and (ii) a table on a scale of 1–10 for scoring the level of negative feelings of the day.

Furthermore, the occupation-based bilateral upper limb training given to the participants in both experimental and control groups was based on the protocol developed by Kim [29]. The protocol allows each patient to be given a more suitable intervention, as patients in different BRS (3–6) should vary in the treatment method among the following: the one involving the hemiplegic hand, the one involving the nonhemiplegic hand, and the one assisted by the therapist. The participants in this study were requested to select and perform via the COPM, five most important occupation-based activities that require the use of both hands. Additionally, for each activity, the patient and therapist prepared any necessary materials for the activity that had been used in the past in advance; therefore, it resembled the one performed at home as much as possible. This was also aimed at facilitating the transfer of the activity to the daily life of each participant. The control group was not given the CBT but the conventional occupational therapy (including neurodevelopmental therapy or exercise therapy based on Bobath approach or proprioceptive neuromuscular facilitation, in-hand manipulation, or dexterity training) in combination with occupation-based bilateral upper limb training.

The results of this study showed that the experimental group of CBT in combination with occupation-based bilateral upper limb training scored significantly less across all tests: ATQ-N, KDS, and STAI-KYZ. According to Yoo et al. [30], the intervention based on cognitive restructuring had an effect of reducing the negative thoughts on the self and the depressive feelings, as CBT focuses on turning the negative automatic thoughts into positive ones. In the randomized controlled study by Gao et al. [31], likewise, depression and anxiety were reported to have significantly decreased in the group of patients with stroke that received CBT when compared to two other groups, which coincided with the results of this study. The experimental group in this study, compared to the control group, showed greater variance across all tests of the upper limb function, while the *p* value of the performance and variance in the COPM were higher. This is presumed to be owing to the intervention for cognitive restructuring performed simultaneously with the behavioral training of muscle relaxation and breathing, in each session after the seventh CBT developed in this study. Ahn et al. [32] reported that, when the intervention combining progressive muscle relaxation and breathing training was given to 18 social workers with chronic pain, positive changes were observed in physical symptoms, depression, and anxiety between the time before and after participating in the program. The study also found significant changes in physiological and neurological parameters, while the effects lasted ≥3 months.

In this study, both groups were given the occupation-based bilateral upper limb training, the result of which was a significant improvement in MFT, MAL, and COPM in both groups. In the study by Kim and Park [6], the experimental group was guided to perform such activities as getting dressed with both hands, using a computer, cooking, and washing dishes, to show a substantial improvement in the upper limb function in comparison to the control group that received the conventional bilateral upper limb training. In M. J. Lee et al.'s [33] study, the experimental group received general occupational therapy involving the use of both hands in addition to the following activities: washing dishes, cutting fruits, and making coffee. Compared to the control group that received only the general occupational therapy twice, the experimental group showed a significant improvement in the performance of daily activities and the upper limb function. Shim and Jung [34] reported that the experimental group that received bilateral upper limb training showed a significant improvement of a higher degree than the control group that received unilateral upper limb training, in terms of the MFT score and the quantity and quality of movement. Kim [29] reported a significant improvement across the satisfaction and performance in COPM and the quantity and quality of movement in MAL, in both the experimental and control groups that received the occupation-based bilateral upper limb training. The experimental group received occupation-based bilateral upper limb training and transcranial electrical stimulation therapy, and the control group received only occupation-based bilateral upper limb training. Both the experimental group and the control group showed improved upper limb function, except that the experimental group to which transcranial electrical stimulation was added showed an increase in the amount of use of the affected side. This suggests that the occupation-based bilateral intervention had a positive effect on the recovery of upper limb function in stroke patients.

Additionally, Arya et al. [35] pointed out the need for a close association between the therapeutic occupations selected by the client and his or her actual daily activities, while Law et al. [36]. reported that, by setting the therapeutic goals themselves, the participants were more actively engaged in the treatment to participate in the occupation with greater commitment, and such active and motivated participation in the training led to increased motor learning and ultimately more outstanding effects in functional recovery than the conventional task-oriented trainings. In the present study, as the target activities were selected based on the participant's opinions regarding the most urgently required tasks, his or her participation was with increased interest and enthusiasm, which improved the detailed hand movements as well as the quantity and quality of movement to ultimately lead to enhanced occupational performance.

The between-group variance after intervention showed a significant difference in ATQ-N, KDS, STAI-KYZ, and COPM but not in MFT or MAL. The lack of a significant difference in MFT or MAL is presumed to be due to the same bilateral upper limb training given to both the experimental and control groups. However, the reason for the greater variance in ATQ-N, KDS, STAI-KYZ, and COPM shown by the experimental group is likely to be due to the effect of the CBT. Murphy et al. [37] conducted a study on patients with osteoarthritis and found a notable beneficial effect of the CBT on pain and fatigue, thus providing a focused discussion on the high level of treatment satisfaction in the participants. In line with this, both the experimental and control groups in this study showed a significant improvement in the two items of COPM, while the variance was increased to a greater degree in the experimental group than in the control group with a particularly large improvement in the satisfaction, which may be attributed to the beneficial effect of CBT including the change towards positive thoughts and feelings and enhanced self-esteem and self-confidence, combined with the previously described positive effect of the occupation-based bilateral upper limb training. This study has several limitations. First, the study period was short at 4 weeks with a small sample size; therefore, the findings in this study cannot be generalized to all patients with stroke. Second, as the participants with hemiplegia on the dominant hand had difficulty writing the daily worksheet of the CBT without the help of a guardian, caretaker, or therapist, their feelings at times were not fully described. Third, a follow-up monitoring to verify the continuity of the intervention effects was not performed. Thus, to complement these limitations, future studies should recruit a larger number of participants and develop CBT programs to allow easy participation without the need of handwriting, and carry out follow-up monitoring to verify whether the intervention provides lasting effects.

The results of this study have the following implications for occupational therapy practice:

As CBT has rarely been used in stroke patients, a novel program developed by the author of this study provided a guideline to the occupational therapists or guardians of stroke patients.

A combined treatment of CBT and occupation-based bilateral upper limb training is predicted to be a useful intervention in occupational therapy for rehabilitation of stroke patients.

## 5. Conclusion

CBT was effective in lowering the levels of depression and anxiety in patients with stroke and increasing satisfaction of occupational performance. The occupation-based bilateral upper limb training was also shown to have a positive impact on upper limb function and occupational performance. Combining CBT with occupation-based bilateral upper limb training will ensure effective treatment for stroke patients with challenges of daily activities due to limited occupational performance and upper limb function along with depression and anxiety.

## Figures and Tables

**Figure 1:** Study process.

**Figure 2:** (a) BRS 3 stage, cleaning the table; (b) BRS 4 stage, washing dishes; (c) BRS 5 stage, setting the table; (d) BRS 6 stage, reading a book.

**Table 1:** Cognitive behavioral therapy.

Stage	Session	Topic	Contents
Initiation	1–3	(i) Introduction to the program and education	(i) Program overview (ii) Information on stroke and hand coordination & education on the use of the hemiplegic upper limb (iii) Education on cognitive behavioral therapy
Development	4–6	(i) To have a positive mindset and build self-confidence	(i) To read positive phrases regarding acceptance (ii) To read poems describing feelings and to highlight favorite words and sentences (iii) To read positive phrases regarding courage and to choose and write down favorite phrases
	7	(i) To learn how to reduce tension by relaxation through breathing	(i) To learn the behavioral techniques of relaxation and breathing ⟶ From session 7 onwards, the relaxation and breathing techniques are practiced at each session
	8	(i) To energize behavior	(i) To record the activity performed at each hour and to evaluate the sense of joy and accomplishment together ⟶ From session 8 onwards, weekly activities are planned together
	9–12	(i) To turn negative thoughts into positive thoughts	(i) To read an autobiography of someone with stroke experience and to make a note of thoughts and resolutions (ii) To draw one's own body while pushing away any negative feelings from the body (iii) To recall a pleasing moment of the day and to record details and the positive feeling of the moment (iv) To think of a pleasant activity and actually perform the activity
	13–17	(i) To improve self-esteem and remember to have a positive mindset	(i) To identify a cognitive distortion and find a solution on one's own (ii) To think of something, one is good at and to write down the thoughts and feelings related to it (iii) To read a negative story and recall the meaning of the story (iv) To remind oneself how valuable he or she is (v) To write a word of advice to another patients with stroke
Termination	18–20	(i) Completion of the program and making a resolution to have a happy life	(i) To learn how to respond to a negative situation (ii) To write about the feelings one had throughout the program (iii) To make a resolution towards one's positive life ahead

**Table 2:** Occupation-based bilateral upper limb training.

Brunnstrom recovery stage (BRS)	Activity	Use of bilateral upper limbs
3	Washing dishes	(i) To use the hemiplegic limb to push down the dishes to fix their positions and to use the nonhemiplegic limb to do the scrubbing
	Dressing	(ii) To use the nonhemiplegic limb to fix the sleeve downwards and to use the hemiplegic limb to stretch into the sleeve
	Cleaning the table	(iii) To use the hemiplegic limb to fix the cloth and to use the nonhemiplegic limb to assist the hemiplegic limb in moving forward and backward while wiping the surface of the table
4	Making a grain powder drink	(i) To use the hemiplegic limb to pull open the refrigerator and to use the nonhemiplegic limb to take out the grain powder
	Washing dishes	(ii) To use the nonhemiplegic limb to hold the sponge and to use the palm of the hemiplegic limb to squeeze out the washing up liquid
	Doing skincare	(iii) To use the hand of the hemiplegic limb to squeeze out the lotion onto the hand of the nonhemiplegic limb and then to use both hands to apply the lotion onto the face
5	Setting the table	(i) To use the nonhemiplegic limb to fix the position of the container and to use the hemiplegic limb to open the cover-style lid of the container
	Washing dishes	(ii) To use the hemiplegic limb to hold the dish and to use the nonhemiplegic limb to do the scrubbing
	Hand washing	(iii) To use both hands to wash a pair of socks by rubbing them together
6	Reading a book	(i) To use the nonhemiplegic limb to fix the position of the book and to use the hemiplegic limb to turn the pages
	Using a computer	(ii) To use both hands to type up a simple document using the keyboard
	Cleaning the house	(iii) To use both hands to wring a wet cloth to squeeze out the water

**Table 3:** General characteristics of participants.

		Experimental group (*n* = 10) *M* (SD)		Control group (*n* = 10) *M* (SD)		*pvalue*
Sex (*n* [%])	M	7	70.0	5	50.0	0.361
	F	3	30.0	5	50.0	
Case type (*n* [%])	Infarction	6	60.0	6	60.0	1.000
	Hemorrhage	4	40.0	4	40.0	
Hemiplegic side (*n* [%])	Right	4	40.0	4	40.0	1.000
	Left	6	60.0	6	60.0	
Average age		61.40 (9.33)^†^		66.60 (8.63)		0.150
Case period, months		4.50 (1.17)		4.60 (1.17)		0.845
BRS		4.40 (0.84)		4.50 (0.85)		0.745

^†^Mean (standard deviation) ∗*p* < 0.05. BRS: Brunnstrom recovery stage.

**Table 4:** Comparison of depression, anxiety, upper limb function, and occupational performance between pretest and posttest and the variance between control and experimental groups.

		Pretest	Posttest	*Z*	*pvalue*	Between-groups	*Z*	*pvalue*
		*M* (SD)	*M* (SD)			*M* (SD)		
ATQ-N	E	98.60 (9.66)^†^	78.20 (9.21)	-2.805	0.005^∗∗^	-21.50 (2.95)	-3.807	*p* < 0.001^∗∗∗^
	C	97.40 (9.77)	96.70 (9.93)	-1.933	0.053	-0.70 (0.94)		

KDS	E	60.50 (8.42)	45.50 (7.09)	-2.816	0.005^∗∗^	-15.00 (1.82)	-3.798	*p* < 0.001^∗∗∗^
	C	59.50 (8.29)	58.30 (8.12)	-1.509	0.131	-1.20 (2.14)		

STAI-KYZ(S)	E	67.70 (7.22)	56.50 (6.67)	-2.829	0.005^∗∗^	-11.20 (2.85)	-3.814	*p* < 0.001^∗∗∗^
	C	68.40 (7.47)	67.20 (7.11)	-1.852	0.064	-0.70 (1.15)		

STAI-KYZ(T)	E	61.80 (8.84)	52.60 (10.28)	-2.692	0.007^∗∗^	-10.10 (1.85)	-3.845	*p* < 0.001^∗∗∗^
	C	62.10 (8.62)	61.40 (8.83)	-1.933	0.053	-0.60 (0.84)		

MFT	E	14.00 (5.61)	19.70 (4.87)	-2.840	0.005^∗∗^	5.70 ± 1.33	-1.538	0.124
	C	14.40 (5.92)	19.20 (5.80)	-2.831	0.005^∗∗^	4.80 ± 1.13		

MAL-AOU	E	60.10 (23.06)	75.00 (23.07)	-2.809	0.005^∗∗^	14.90 ± 3.14	-1.227	0.220
	C	61.60 (21.72)	74.90 (22.92)	-2.814	0.005^∗∗^	13.30 ± 2.21		

MAL-QOM	E	58.50 (23.61)	68.50 (24.50)	-2.831	0.005^∗∗^	10.00 ± 1.82	-1.500	0.134
	C	59.80 (22.65)	68.30 (23.59)	-2.814	0.005^∗∗^	8.50 ± 2.06		

COPM-P	E	3.10 (1.36)	6.78 (1.40)	-2.814	0.003^∗∗^	3.68 ± 0.70	-3.971	*p* < 0.001^∗∗∗^
	C	3.20 (1.51)	5.22 (1.50)	-3.051	0.005^∗∗^	2.02 ± 0.06		

COPM-S	E	1.92 (0.97)	6.30 (1.65)	-2.818	0.003^∗∗^	4.38 ± 0.89	-3.845	*p* < 0.001^∗∗∗^
	C	2.80 (1.25)	4.84 (1.22)	-2.972	0.005^∗∗^	2.04 ± 0.08		

∗*p* < 0.05, ∗∗*p* < 0.01, and ∗∗∗*p* < 0.001. E: experimental group; C: control group; ATQ-N: Automatic Thoughts Questionnaire-Negative; KDS: Korean Depression Scale; STAI-KYZ: State Trait Anxiety Inventory-Korean YZ; MFT: Manual Function Test; MAL: Motor Activity Log; COPM: Canadian Occupational Performance Measure.

## Data Availability

(1) The data used to support the findings of this study were supplied under license and so cannot be made freely available. Requests for access to these data should be made thdms987@naver.com. (2) The data used to support the findings of this study are currently under embargo while the research findings are commercialized. Requests for data, 12 months after publication of this article, will be considered by the corresponding author. (3) The data used to support the findings of this study may be released upon application to Choi, who can be contacted at thdms987@naver.com.
